# Qijiaoshengbai Capsule for Leukopenia: A Systematic Review and Meta-Analysis of Randomized Controlled Trials

**DOI:** 10.1155/2021/1972981

**Published:** 2021-10-23

**Authors:** Hongfang Fu, Yilan Wang, Haoyue Feng, Yang Zhang, Xiaoyu Hu

**Affiliations:** ^1^Hospital of Chengdu University of Traditional Chinese Medicine, Chengdu 610072, Sichuan Province, China; ^2^School of Clinical Medicine, Chengdu University of Traditional Chinese Medicine, Chengdu 611137, Sichuan Province, China

## Abstract

Qijiaoshengbai capsule (QJSBC) is a type of proprietary Chinese medicine, which is an effective treatment for leukopenia in clinical practice. The purpose of this study is to evaluate the efficacy of QJSBC in improving specific clinical indicators, in patients with leukopenia of various origins. A total of seven electronic databases were searched, up until an end date of April 30, 2021, and a selection of clinical indicators was noted. The primary indicators of concern were related to blood: white blood cells (WBC). Secondary indicators were hemoglobin (Hb), platelets (PLT), neutrophils (NEU), bone marrow suppression rate (BMSR), and effective rate (ER). The methodological quality of the included trials was analyzed using a risk of bias assessment, as per the Cochrane Manual. The meta-analysis was performed using RevMan 5.4. *Results*. Twenty-four randomized controlled trials involving a total of 2,692 participants were included in this review. We found that QJSBC had a positive effect on increasing WBC, HB, PLT, and NEU and improving BMSR and ER. *Conclusion*. When compared with conventional chemotherapy (CC), conventional radiotherapy (CR), combined chemotherapy and radiotherapy (CC + CR), or conventional treatment (CT), the use of QJSBC combined therapy can effectively improve the clinical outcome for patients with leukopenia. However, a larger sample size and a more standardized, high-quality study are required to validate these results.

## 1. Introduction

Leukopenia is a common blood disease with an incidence of 12.4% [1], in which the peripheral blood leukocyte count is less than 4 × 10^9^/L [2]. Patients with mild symptoms may experience fatigue, dizziness, palpitations, loss of appetite, low fever, and chills. In addition, on top of this, patients with severe symptoms may also suffer from the common upper respiratory tract, urinary tract, and secondary infections, with their condition characterized by repeated attacks and difficult recovery [3, 4]. The clinical etiology of leukopenia is complicated, with drug-induced leukopenia being the most common [5]. Examples include radiotherapy and chemotherapy drugs and antithyroid, psychiatric, and antihepatitis medications [6]. Leukopenia is seen in up to 70% of tumor patients after chemotherapy [7]. Severe bone marrow suppression (BMS) caused by chemotherapeutic drugs is the main reason that cancer patients are not able to continue chemotherapy, as it seriously affects the efficacy of treatment, prolongs the length of hospital stays, increases the cost to patients, and in some cases can even be fatal [8]. One study [9] showed that patients aged 41–70 years were most likely to be diagnosed with leukopenia. A possible reason for this may be that leukopenia is related to a change of pharmacokinetics in this age group; however, it should be noted that this is also consistent with the age distribution of cancer patients in China (showing a peak between 45 and 74 years of age). At present, granulocyte colony-stimulating factor (G-CSF) is commonly used in the treatment of leukopenia [10]. However, the high price of this drug creates a heavy economic burden on patients, and with common side effects such as skeletal muscle pain, low fever, and increased tumor risk, it is not optimal [11].

In China, traditional Chinese medicine (TCM) has shown good safety and efficacy in the prevention and treatment of leukopenia and BMS. Various prevention and treatment methods used include a medicated diet, acupuncture, moxibustion, and Chinese herbal medicine and they all have wide application and can be implemented in various forms [12–15]. Capsules of Qijiaoshengbai (QJSBC) is a proprietary Chinese medicine used in the treatment of leukopenia of various etiologies (Approval No. Z20025027). It is composed of seven authentic Guizhou herbs: Chinese jujube (da zao), blood ginseng (xue ren shen), *Astragalus membranaceus* (huang qi), Colla corii asini (e jiao), *Angelica sinensis* (dang gui), *Sophora flavescens* (ku shen), and *Epimedium* (yin yang huo) [16]. Since its launch, QJSBC has become one of the more commonly used Chinese patent medicines used in China to treat leukopenia. Studies have found that QJSBC has antitumor properties; it improves immunity, increases WBC and PLT counts, inhibits oxidation, and improves tissue perfusion [17].

In 2015, a systematic review and meta-analysis of QJSBC in the treatment of leukopenia was published in China [4]. However, that paper is now outdated as it does not include more recent literature published between 2015 and 2021, and there are other flaws. In this study, we evaluate the efficacy of QJSBC in preventing leukopenia and alleviating BMS via rigorous systematic evaluation and meta-analysis, to facilitate evidence-based medicine for clinical treatment.

## 2. Methods

### 2.1. Search Strategy

The systematic review and meta-analysis was based on the Preferred Reported Items for Systematic Reviews and Meta-Analysis (PRISMA) statement [18]. The following seven databases were searched from their inception up until April 30, 2021: PubMed, Embase, Cochrane Library, China National Knowledge Infrastructure (CNKI) database, Wanfang Data Knowledge Service Platform, the VIP information resource integration service platform (cqVIP), and China Biology Medicine Disc (Sino Med). The keywords used to search for randomized controlled trials (RCTs) were “qijiaoshengbai” OR “qi-jiao-sheng-bai” OR “qijiaoshengbaijiaonang” OR “qijiaoshengbai capsule,” “leukopenia” OR “hypoleucocytosis” OR “hypolekocytosis” OR “marrow suppression” OR “bone marrow suppression” OR “bone marrow suppression rate,” and “clinical trial” OR “randomized controlled trial.” All the citations were searched and screened by two authors to reduce the risk of leaving out any relevant references. There was no limit imposed on the language of the search results.

### 2.2. Selection Criteria

#### 2.2.1. The Review Included RCTs That Met the Criteria Listed below

1. Patients had an established diagnosis of leukopenia;
2. The treatment group was treated with QJSBC or QJSBC combined with other methods, while the control group was treated with non-QJSBC;
3. Outcome indicators included WBC, PLT, Hb, NEU, BMSR (with evaluation criteria referring to the WTO Anticancer Drug Classification Standard) [19] and ER.

There were no limitations in terms of gender, race, or country.

#### 2.2.2. Literature Was Excluded If It Met the following Criteria

Duplicate studies, review articles, animal experiments, systematic evaluation, graduation papers, retrospective, cross-sectional studies, and conference abstracts.

### 2.3. Study Selection and Data Extraction

Two researchers selected the literature used in our study according to the inclusion and exclusion criteria after independently reading the title, abstract, and full text of each study. A data extraction template was created to extract the following information: first author, publication year, number of participants sampled, age, gender, intervention method, and course of treatment. Discrepancies between the two authors were resolved through discussion.

### 2.4. Quality Assessment and Statistical Analysis

The methodological quality of the selected trials was assessed according to the Cochrane Collaboration's tool [20]. Review Manager Version 5.4 was used to create a forest plot and conduct subgroup analysis. Relative risk (RR) was used for enumeration data; mean difference (MD) or standardized mean difference (SMD) was used for measurement data; and the range was expressed as the 95% confidence intervals (CI). Statistical heterogeneity was considered significant when *p* < 0.1 and *I*^2^ >50%, and in this case, a random effects model was used to calculate the effect size. When *p* < 0.1 and *I*^2^ <50%, the studies included were considered homogeneous and a fixed effects model was applied. Sensitivity analysis was conducted to test whether the result was robust by excluding the studies individually and comparing the effects of the remaining studies with the total effects of all the studies. Publication bias was assessed using a funnel plot analysis.

## 3. Results

### 3.1. Study Selection

From a total of 200 potentially related studies found during our initial search, 98 records were evaluated after the exclusion of 102 duplicates. Based on the titles and abstracts, an additional 52 studies were excluded as they were either a review, systematic evaluation, animal experiment, graduation paper, or conference abstract. This left 46 full-text articles, from which we excluded 22 trials because they were not randomized, the data were not reliable, or the outcomes measured did not meet our requirements. Therefore, a final total of 24 studies [21–44], including 1,424 patients in the experimental group and 1,268 patients in the control group, were selected for this study. A schematic of the selection process is shown in Figure 1.

### 3.2. Study Characteristics

Table 1 presents the main characteristics of the included trials. In total, 24 studies were selected, with 2,692 participants ranging in age from 14 to 81 years. The sample size varied widely between studies (from 52 to 297 participants), and all were conducted in China and published between 2013 and 2021. Each article consisted of QJSBC treatment in the experimental group and non-QJSBC treatment in the control group. Our control group included 13 studies [21–24, 29, 30, 32–35, 39, 40, 42] using CC, 2 studies [25, 26] using CR, 2 studies [27, 31] using CC + CR, 2 studies [22, 32] using CC + ADLC, and 7 studies [28, 36–38, 41, 43, 44] using CT. Overall, 21 studies [21–23, 25–30, 32–38, 40–44] reported WBC, 10 studies [21, 23, 27, 29, 30, 32–34, 40, 42] reported Hb, 13 studies [21, 23, 27, 29, 30, 32–35, 40–43] reported PLT, 7 studies [22, 23, 32, 33, 35, 36, 43] reported NEU, 8 studies [24–27, 31, 33, 35, 39] reported BMSR, and 4 studies [21, 37, 40, 42] reported ER.

### 3.3. Methodological Quality

Two reviewers independently conducted a risk of bias assessment using the Cochrane Collaboration's tool. Using this method, the risk of bias of each trial was assessed based on seven components: random sequence generation (selection bias), allocation concealment (selection bias), blinding of participants and personnel (performance bias), blinding of outcome assessment (detection bias), incomplete outcome data (attrition bias), selective reporting (reporting bias), and other bias. The methodological quality assessment for each of the relevant studies is shown in Figures 2 and 3. Of these, two trials [22, 32] referred to blinding and allocation concealment, and three studies [22, 24, 32] reported the withdrawal of participants from the study, which resulted in incomplete data. No selective reporting or other biases were found. Any discrepancies were resolved by discussion among all reviewers.

### 3.4. Outcomes of the Indicators

#### 3.4.1. WBC Counts

A total of 21 research trials [21–23, 25–30, 32–38, 40–44] with 2155 patients evaluated the effect of QJSBC on WBC, with 1162 patients in the QJSBC treatment group and 993 patients as control. A meta-analysis of these results revealed that, compared to the control group, treatment with QJSBC significantly improved WBC counts (MD = 1.08, 95% CI: [0.90, 1.26] , *p* < 0.00001; heterogeneity: *p* < 0.00001, *I*^2^ = 96%, random effects model) (Figure 4). Subsequently, a subgroup analysis was performed based on disease type, control group treatment, and treatment duration (Figures 5(a)–5(c)). The analysis of the disease type provided the following results for the subgroups “tumor-associated leukopenia” (MD = 1.17; 95% CI [0.94, 1.40]), and “nontumor-associated leukopenia” (MD = 0.91; 95% CI [0.52, 1.29]). The analysis based on the treatment plan of the control group provided the following results: “CC” subgroup (MD = 1.08; 95% CI [0.86, 1.31]); “CR” subgroup (MD = 1.22; 95% CI [1.05, 1.38]); “CC + ADLC/CC + CR” subgroup (MD = 2.34; 95% CI [−0.43, 5.10]); and “CT” subgroup (MD = 0.84; 95% CI [0.49, 1.18]). Finally, an analysis of the postmortem subgroup was performed according to the duration of treatment, showing “treatment duration less than 1 month” subgroup (MD = 0.88; 95% CI [0.63, 1.13]); “treatment duration longer than 1 month” subgroup (MD = 1.25; 95% CI [1.03, 1.47]); and “treatment duration unclear” subgroup (MD = 1.82; 95% CI [0.59, 3.05]). Based on these results, we concluded that the source of the heterogeneity of WBC counts may be related to the treatment time of the disease, whilst being independent of the disease type and treatment plan of the control group. According to the results of the funnel plot test, no publication bias was evident (Figure 6).

#### 3.4.2. Hb Counts

The effect of QJSBC on Hb count was reported in 10 trials [21, 23, 27, 29, 30, 32–34, 40, 42], involving a total of 955 patients. The pooled results suggest that QJSBC might increase Hb counts of patients in the QJSBC treatment group (MD = 18.12; 95% CI [13.68, 22.56], *p*=0.00001), with high heterogeneity (*p* < 0.00001, *I*^2^ = 87%, random effects model) (Figure 7). A subgroup analysis was conducted according to the treatment plan of the control group with the following results: “CC” subgroup (MD = 20.53; 95% CI [16.27, 24.80]) and “CC + ADLC/CC + CR” subgroup (MD = 8.82; 95% CI [4.11, 13.53]) (Figure 8). Based on these results, we conclude that the source of heterogeneity in Hb counts may be related to the treatment plan of the control group. Since all the studies in this group were related to leukopenia of tumor-related diseases, subgroup analysis of disease types was not conducted. The funnel plot suggested a low probability of publication bias (Figure 9).

#### 3.4.3. PLT Counts

PLT count was reported in 13 studies [21, 23, 27, 29, 30, 32–35, 40–43], involving a total of 1200 patients. All studies demonstrated the therapeutic effect of QJSBC with high heterogeneity (MD = 45.80, 95% CI [29.00, 62.60], *p* < 0.00001 heterogeneity: *p* < 0.00001, *I*^2^ = 98%, random effects model) (Figure 10). A subgroup analysis was performed based on disease type and the following results were obtained, as shown in Figure 11(a): “tumor-associated leukopenia” subgroup (MD = 46.30; 95% CI [28.81, 63.79]) and “nontumor-associated leukopenia” subgroup (MD = 39.00; 95% CI [12.64, 65.36]). A subgroup analysis according to the treatment plan of the control group revealed “CC” subgroup (MD = 54.32; 95% CI [33.69, 74.94]); “CC + ADLC/CC + CR” subgroup (MD = −3.41; 95% CI [−40.08, 33.26]); and “CT” subgroup (MD = 53.72; 95% CI [33.12, 74.33]) (Figure 11(b)). According to these results, the source of heterogeneity of PLT counts may be related to the treatment plan of the control group and is independent of the disease type. The funnel plot was asymmetric, which suggested that there was a publication bias between the results of PLT counts (Figure 12).

#### 3.4.4. NEU Counts

The impact of the addition of QJSBC on NEU levels was assessed in 7 studies [22, 23, 32, 33, 35, 36, 43]. The results showed that, compared with the control group, the group treated with QJSBC had significantly increased NEU counts (MD = 0.59, 95% CI [0.15, 1.03], *p*=0.009; heterogeneity: *p* < 0.00001, *I*^2^ = 89%, random effects model) (Figure 13). As shown in Figure 14(a), a subgroup analysis based on disease type showed “tumor-associated leukopenia” (MD = 0.44; 95% CI [−0.09, 0.97]) and “nontumor-associated leukopenia” subgroup (MD = 0.93; 95% CI [0.05, 1.81]). A subgroup analysis conducted according to the treatment plan of the control group gave the following results: “CC” subgroup (MD = 0.75; 95% CI [0.07, 1.43]); “CC + ADLC” subgroup (MD = −0.28; 95% CI [−0.94, 0.39]); and “CT” subgroup (MD = 0.93; 95% CI [0.05, 1.81]) (Figure 14(b)). According to these results, the heterogeneity of the NEU counts may be related to the treatment plan of the control group and may be independent of the disease type. Because the number of RCTs included in NEU counts was less than 10, there was no funnel chart analysis for this part of data.

#### 3.4.5. Bone Marrow Suppression Rate

BMSR were mentioned in 8 of the trials [24–27, 31, 33, 35, 39]. Based on our assessment, when compared with controls, the use of QJSBC for treatment may reduce the occurrence of bone marrow suppression (RR = 0.16, 95% CI [0.12, 0.22], *p* < 0.00001; heterogeneity: *p*=0.27, *I*^2^ = 20%, fixed effects model) and there was no funnel chart analysis (Figure 15).

#### 3.4.6. Effective Rate

The ER was mentioned in 4 studies [21, 37, 40, 42], with a total of 287 patients. There was an absence of substantial heterogeneity (RR = 6.56, 95% CI [2.79, 15.40], *p* < 0.0001, heterogeneity: *p*=0.95, *I*^2^ = 0%, fixed effects model) (Figure 16). The meta-analysis results revealed that compared to controls, QJSBC treatment significantly improved the ER of patients and there was no funnel chart analysis for this part of data.

### 3.5. Sensitivity Analysis

A sensitivity analysis was used to evaluate the robustness of the combined results. The analysis showed that no individual study had a significant impact on the overall results. Based on the sensitivity analysis, the combined effect size of WBC counts, Hb counts, PLT counts, NEU counts, BMSR, and ER was stable.

## 4. Discussion

Leukopenia, a common blood disease with a high incidence, is also a common clinical disease symptom and reacts adversely to medication [45]. Clinically, leukopenia causes recurrent infection, especially in tumor patients, which is not conducive to further radiation and chemotherapy. Despite its rapid response, G-CSF, although commonly used, is not suitable for long-term use in all patients due to its short duration of efficacy, high cost, and the increased risk of secondary malignancy.

According to TCM theory, leukopenia belongs to the category of “deficiency of fatigue” (Xu lao) [46], with most patients having a deficiency of both Qi and blood. Thus, QJSBC is used for treatment as it has the effect of enriching blood and replenishing Qi [47]. TCM doctors tend to use proprietary Chinese medicines flexibly based on TCM theories, which often results in a lack of adequate evidence-based support for the treatment of diseases with proprietary Chinese medicines.

According to the current results from randomized controlled trials, QJSBC combined with western medicine can help to increase the count of WBC, Hb, PLT, and NEU; reduce the BMSR; and improve the ER. Many of the published studies [24, 31, 39] did not include all of these indicators, all of which show the advantage of QJSBC in improving the BMSR. In addition, the proprietary Chinese medicine QJSBC is generally safe, with no studies finding that it caused serious adverse events. A subgroup analysis of outcome indicators with heterogeneity was conducted to find the source of the heterogeneity. We found that the heterogeneity may be related to the type of disease, the treatment plan, and the duration of treatment. The funnel plot of PLT counts suggested that there was a publication bias. Sensitivity analysis showed that the results for WBC, Hb, PLT, NEU, BMSR, and ER were robust for all changes.

A meta-analysis [4] published in 2015 examined the efficacy of QJSBC. However, flaws exist in this article. First, the authors searched a small number of databases and second, the authors used inappropriate methods when sorting the data and interpreting the results. We consider the results of the 2015 article misleading and suggest that the methods used in our study are more appropriate and effective, giving more reliable results.

Systematic reviews and meta-analyses are at the top of the hierarchy of clinical evidence, and we have used this approach to determine the efficacy of QJSBC on patients with leukopenia, aiming to provide an up-to-date clinical evaluation of treatment with QJSBC. This effective and low-cost Chinese patented medicine has the potential to benefit an increasing number of leukopenia patients around the world, helping to somewhat reduce the economic burden on patients, their families, and society.

## 5. Limitations

Throughout the study, we have taken care of interpreting our results carefully; however, there are some limitations to consider. (1) All the included studies were published in Chinese and all the patients were Chinese, so it is not clear whether the results apply to patients from other regions. (2) There were only two high-quality, multicenter, randomized, double-blind studies. The inclusion of other studies that not meeting these criteria resulted in a lack of convincing results. The overall methods included in these studies were of low quality due to incomplete data collection, and deficiencies in study design. More large-sample, multicenter, high-quality randomized controlled trials are needed for validation. (3) The fact that only 1 out of 24 trials was publicly registered means we are not able to rule out the possibility of publication bias.

## 6. Conclusion

In conclusion, this systematic review and meta-analysis evaluated the effect of QJSBC for treating leukopenia in cancer patients and comprehensively analyzed the results of randomized controlled trials published between 2013 and 2021. The systematic review and meta-analysis showed that QJSBC when compared with a non-QJSBC control group had more beneficial effects on several clinical indicators (WBC, Hb, PLT, NEU, BMSR, and ER). Although QJSBC was effective in treating leucopenia in all 24 studies, larger sample sizes and higher-quality randomized controlled trials are needed to reduce study heterogeneity and validate these findings.

## Figures and Tables

**Figure 1:** Flow diagram of search and selection process.

**Figure 2:** Risk of bias.

**Figure 3:** Risk of bias.

**Figure 4:** Forest plot for WBC.

**Figure 5:** Forest plot of WBC subgroup analysis: (a) disease type, (b) control group treatment, (c) treatment duration.

**Figure 6:** Funnel plot for the publication bias of WBC.

**Figure 7:** Forest plot of Hb.

**Figure 8:** Forest plot of Hb subgroup analysis.

**Figure 9:** Funnel plot for the publication bias of Hb.

**Figure 10:** Forest plot of PLT.

**Figure 11:** Forest plot of PLT subgroup analysis: (a) disease type and (b) control group treatment.

**Figure 12:** Funnel plot for the publication bias of PLT.

**Figure 13:** Forest plot of NEU.

**Figure 14:** Forest plot of NEU subgroup analysis: (a) disease type and (b) control group treatment.

**Figure 15:** Forest plot of BMSR.

**Figure 16:** Forest plot of ER.

**Table 1:** Characteristics of the included trials.

Author/year	Number of subjects		Male/female		Age : mean ± SD		Intervention		Treatment duration
	E	C	E	C	E	C	E	C	
Chong Wang, 2020	38	38	22/16	21/17	51.00 ± 3.50	50.50 ± 3.00	QJSBC + CC	CC	NR
Tongde Zhao, 2020	192	95	77/115	38/57	54.70 ± 10.66	55.24 ± 10.60	QJSBC + CC	CC + ADLC	20 d
Jing Xie, 2015	72	68	48/24	42/26	60.5 ± 4.2	57 ± 3.5	QJSBC + CC	CC	18 w
Li Zhang, 2017	157	140	89/73	83/79	37.13 ± 12.13	36.95 ± 11.56	QJSBC + CC	CC	12 w
Rongmei Ding, 2016	70	70	37/33	38/32	50–72	51–73	QJSBC + CR	CR	4-5 w
Bo Chen, 2017	51	51	30/21	33/18	55.3 ± 4.8	56.6 ± 4.7	QJSBC + CR	CR + CT	4 w
Chi Zhang, 2018	75	75	41/34	43/32	37.01 ± 5.58	36.78 ± 5.47	QJSBC + CC	CC	6 w
Fan Huang, 2020	68	68	36/32	41/27	48.41 ± 5.91	51.62 ± 6.75	QJSBC + CC + CR	CC + CR	NR
Hong Lin, 2015	60	59	32/28	29/30	40 ± 10	41 ± 10	QJSBC + CT	CT	4 w
Zhenguo Song, 2018	50	50	28/22	30/20	51.3 ± 4.2	51.7 ± 3.9	QJSBC + CC	CC	8 w
Yuan Gao, 2013	27	25	17/10	13/12	36–70	32–70	QJSBC + CC	CC	12 w
Xinhu Wu, 2013	30	60	17/13	37/23	26–75	28–76	QJSBC + CC + CR + CT	CC + CR + CT	NR
Liyuan Lv, 2020	82	34	77/32	38/14	58.64 ± 9.66	57.77 ± 10.37	QJSBC + CC + ADLC	CC + ADLC	20 d
Shengping Li, 2019	32	32	18/14	17/15	64.34 ± 10.03	63.16 ± 8.14	QJSBC + CC	CC	21 d
Shengtao Fan, 2018	30	28	15/15	14/14	49.5 ± 5.6	49.5 ± 5.7	QJSBC + CC	CC	NR
Wei Zheng, 2013	42	41	NR	NR	55.2 ± 5.7	55.2 ± 5.7	QJSBC + CC	CC	30 d
Hong Yu, 2019	30	30	17/13	16/14	45.16 ± 10.13	45.33 ± 10.29	QJSBC + CC	CC	3 w
Yi Zhang, 2013	46	40	28/18	26/14	34 ± 14	29 ± 16	QJSBC + CT	CT	8 w
Cai Liu, 2017	34	34	21/13	22/12	38.6 ± 1.2	38.9 ± 1.3	QJSBC + CT	CT	4 w
Jingjing Cheng, 2013	48	50	26/22	24/26	36.0 ± 3.3	39.0 ± 2.7	QJSBC + CT	CT	1 m
Liyun Guan, 2015	50	50	64/36	64/36	39–69	39–69	QJSBC + CT	CT	28 d
Hui Liu, 2016	43	42	22/21	20/22	56.3 ± 10.2	56.5 ± 10.1	QJSBC + CC	CC	30 d
Ping Liu, 2013	47	38	29/18	21/17	14–60	16–56	QJSBC + CT	CT	4 w
Yuzhi Yang, 2013	50	50	NR	NR	21∼55	21∼55	QJSBC + CT	CT	4 w

QJSBC = Qi Jiao Sheng Bai Capsule, ADLC = An Duo Lin Capsule, CC = conventional chemotherapy, CT = conventional treatment, CR = conventional radiotherapy), *m* = month, w = weeks, d = days, NR = not reported.
